# Incidence and mortality of multiple myeloma in China, 2006–2016: an analysis of the Global Burden of Disease Study 2016

**DOI:** 10.1186/s13045-019-0807-5

**Published:** 2019-12-10

**Authors:** Jiangmei Liu, Weiping Liu, Lan Mi, Xinying Zeng, Cai Cai, Jun Ma, Lijun Wang, Union for China Lymphoma Investigators of the Chinese Society of Clinical Oncology, Union for China Leukemia Investigators of the Chinese Society of Clinical Oncology

**Affiliations:** 1 National Center for Chronic and Noncommunicable Disease Control and Prevention, Chinese Center for Disease Control and Prevention, Beijing, China; 2 Key Laboratory of Carcinogenesis and Translational Research (Ministry of Education), Department of Lymphoma, Peking University Cancer Hospital & Institute, Beijing, China; 3 Beijing Institute of Survey and Mapping, Beijing Municipal Key Laboratory of Urban Spatial Information Engineering, Beijing, China; 4 Harbin Institute of Hematology & Oncology, Harbin, China

**Keywords:** Multiple myeloma, Incidence, Mortality, Epidemiology

## Abstract

**Background:**

The accurate information about burden of multiple myeloma (MM) at national and provincial level remains unknown in China.

**Methods:**

Following the general analytical strategy used in GBD 2016, the age-, sex-, and province-specific incidence and mortality in China were analyzed. Trends in the incidence and mortality from 2006 to 2016 were evaluated.

**Results:**

It was estimated that there were 16,500 new cases and 10,300 deaths of multiple myeloma in China in 2016. The age-standardized incidence rates (ASIR) and mortality rates (ASMR) per 100,000 population were 1.03 (95% UI, 0.88–1.17) and 0.67 (95% UI, 0.59–0.77) in 2016. Males had higher incidence and mortality rates than females in all age groups. An upward trend with age in incidence and mortality was observed. Higher incidence and mortality rates clustered in the developed provinces. The incidence of MM in China increased significantly from 2006 to 2016, while the mortality increased from 2006 to 2014, and remained stable from 2014 to 2016.

**Conclusion:**

The burden of MM showed a heterogeneous pattern in China, which highlighted the need of tailored disease prevention and control strategies in both national and provincial levels.

## Background

Multiple myeloma (MM) is the second most frequent hematological disease worldwide [1]. In 2016, the incident cases of MM in the most populous countries were 139,000 with the rank of 26 among all cancers, and death number was 98,000 with the rank of 22 among all cancers [2]. According to the statistics of GLOBOCAN 2018, MM accounted for 0.9% of all new cancer cases and 1.1% of all cancer deaths worldwide in 2018 [3]. A recent study estimated that there were 52,000 deaths associated with lymphoma and myeloma and the age-standardized mortality rate was 3.74 per 100,000 population in China in 2017.While the age-standardized mortality rate for lymphoma and myeloma worldwide was 2.60 per 100,000 population. Moreover, the mortality rates of lymphoma and myeloma increased annually by 4.5% from 2004 to 2016 in China [4].

Until now, accurate epidemiologic study of MM based on national and province level has not been conducted in China. In this analysis, we sought to determine the incidence and mortality of multiple myeloma in China in 2016 and analyze temporal trends from 2006 to 2016.

## Methods

### Data sources

Details of the methodology used in the Global Burden of Disease 2016 (GBD 2016) study have been explained in previous studies [5–7]. Briefly, the GBD study provides a highly standardized approach to dealing with the multiple measurement challenges in the cause of death assessment and provided a comprehensive assessment of age-specific, sex-specific, all-cause, and cause-specific mortality rates for all major diseases and injuries for 195 countries and territories from 1980 to 2016. The present study focused on the burden of multiple myeloma nationally and 33 province-level administrative units in China, including Hong Kong and Macao Special Administrative Regions, all of which we refer to as provinces in this study. International Classification of Diseases-10 (ICD-10) codes were used to represent multiple myeloma (C88-C90.32).

The main data sources GBD used for multiple myeloma mortality estimates come from the disease surveillance points system and the cause of death reporting system from Chinese Center for Disease Control and Prevention. All data sources that were used in GBD study were mapped to the GBD standard GBD ICD-10 cause list [5]. The underreporting adjustment and garbage code redistribution were applied for more accurate estimates of multiple myeloma mortality. In GBD 2016, causes that cannot be underlying causes of death (termed garbage codes) are reassigned to causes that can be underlying causes of death. According to the regional variations of data quality across county, different underreporting rates were used to adjust the estimation of mortality. We used the GBD 2016 standard population for computing age-standardized rates. We generated a 95% uncertainty interval (UI) for all quantities reported in the article.

For GBD 2016, we used DisMod-MR 2.1, a Bayesian meta-regression tool, as the main method of estimation, ensuring consistency between incidence, prevalence, remission, and cause of death rates for each condition. We used a compartmental model structure with a series of differential equations that synthesize spares and heterogeneous epidemiological data, including systematic reviews, gray literature sources, and survey data. Detailed descriptions of the modeling strategy for incidence estimation and validation have been published elsewhere [7]. The number of incidence and age-standardized incidence rate of multiple myeloma and 95% UI were reported.

### Statistical analysis

Temporal trends in incidence and mortality rates from 2006 to 2016 were examined by IBM SPSS Statistics for Windows (Version 21.0; IBM Corp) and fitting joinpoint models (version 4.6.0.0; National Cancer Institute). The trends were expressed as annual percentage changes (APCs), and Z tests were used to assess whether the APCs were significantly different from zero. In describing trends, the terms “increase” and “decrease” would be used when the slope of the trend was statistically significant; otherwise, the term “stable” was used. Statistical significance was assessed at the 0.05 level, and all hypothesis tests were two-sided.

## Results

### Incidence and mortality of multiple myeloma in China, 2016

It was estimated that there were 16,500 new cases and 10,300 deaths of multiple myeloma in China in 2016. The age-standardized incidence rates (ASIR) and age-standardized mortality rates (ASMR) per 100,000 population were 1.03 (95% UI, 0.88–1.17) and 0.67 (95% UI, 0.59–0.77) in 2016. After the age of 15 years, the incidence and mortality rates increased steadily with age, and higher incidence and mortality rates of multiple myeloma were seen in the individuals over 60 years (Table 1, Fig. 1). Both ASIR and ASMR had an upward trend with age, and the peak occurred at the age group of 90–94 years. In addition, 1.5–2-folds sex-specific difference of ASIR and ASMR was observed; males were consistently higher than females.

**Table 1:** Incidence and mortality rates of multiple myeloma by age and gender in 2016 (per 100,000 population)

Age groups	Incidence rates			Mortality rates		
	Both	Male	Female	Both	Male	Female
0-	0.00	0.00	0.00	0.00	0.00	0.00
1-	0.00	0.00	0.00	0.00	0.00	0.00
5-	0.00	0.00	0.00	0.00	0.00	0.00
10-	0.00	0.00	0.00	0.00	0.00	0.00
15-	0.18 (0.11–0.22)	0.24 (0.12–0.30)	0.12 (0.07–0.14)	0.09 (0.05–0.10)	0.11 (0.06–0.13)	0.06 (0.04–0.07)
20-	0.22 (0.14–0.26)	0.27 (0.14–0.33)	0.18 (0.10–0.22)	0.09 (0.06–0.11)	0.10 (0.05–0.12)	0.08 (0.05–0.10)
25-	0.29 (0.18–0.34)	0.39 (0.21–0.47)	0.18 (0.11–0.22)	0.10 (0.06–0.11)	0.12 (0.07–0.14)	0.07 (0.04–0.08)
30-	0.25 (0.17–0.30)	0.34 (0.21–0.42)	0.16 (0.09–0.20)	0.10 (0.07–0.11)	0.12 (0.08–0.14)	0.07 (0.04–0.08)
35-	0.31 (0.23–0.37)	0.42 (0.28–0.52)	0.20 (0.12–0.24)	0.14 (0.11–0.15)	0.17 (0.12–0.21)	0.10 (0.07–0.12)
40-	0.51 (0.41–0.59)	0.66 (0.48–0.79)	0.36 (0.24–0.44)	0.26 (0.21–0.29)	0.31 (0.24–0.38)	0.20 (0.14–0.25)
45-	0.87 (0.70–0.97)	1.08 (0.79–1.33)	0.64 (0.47–0.75)	0.44 (0.37–0.49)	0.51 (0.39–0.64)	0.37 (0.27–0.43)
50-	1.71 (1.44–1.99)	2.08 (1.56–2.67)	1.32 (0.99–1.64)	0.88 (0.77–1.02)	0.99 (0.77–1.27)	0.76 (0.57–0.92)
55-	2.44 (2.03–2.96)	3.15 (2.33–4.00)	1.71 (1.36–2.19)	1.33 (1.14–1.59)	1.62 (1.23–2.08)	1.04 (0.84–1.33)
60-	3.62 (3.00–4.28)	4.63 (3.36–5.77)	2.60 (2.08–3.17)	2.19 (1.87–2.59)	2.60 (1.96–3.36)	1.77 (1.45–2.15)
65-	4.60 (3.92–5.47)	5.68 (4.25–7.20)	3.53 (2.88–4.54)	3.11 (2.71–3.75)	3.52 (2.74–4.58)	2.71 (2.22–3.44)
70-	5.36 (4.42–6.29)	7.00 (5.16–8.67)	3.76 (3.00–5.03)	3.83 (3.27–4.50)	4.63 (3.58–5.81)	3.05 (2.44–4.06)
75-	5.71 (4.63–6.57)	7.62 (5.48–9.40)	3.96 (3.20–4.92)	4.45 (3.67–5.18)	5.40 (4.03–7.02)	3.58 (2.91–4.45)
80-	4.01 (3.30–4.66)	5.43 (3.83–6.77)	2.79 (2.27–3.45)	4.11 (3.45–4.91)	5.39 (3.97–6.92)	3.01 (2.42–3.73)
85-	4.65 (3.94–5.70)	6.37 (4.72–8.53)	3.50 (2.95–4.40)	4.68 (4.03–5.79)	6.14 (4.70–8.38)	3.69 (3.05–4.60)
90-	7.07 (6.31–8.83)	9.18 (7.34–13.02)	6.03 (5.21–7.70)	6.96 (6.20–8.80)	8.56 (7.00–12.29)	6.17 (5.30–7.75)
95-	6.43 (5.70–8.43)	9.14 (7.59–13.33)	5.48 (4.74–7.26)	6.38 (5.62–8.42)	8.50 (7.16–12.70)	5.65 (4.88–7.49)

Data in parentheses are 95% uncertainty intervals

**Fig. 1:** Age-specific incidence and mortality rates of multiple myeloma by sex in China, 2016

### Provincial-level incidence and mortality of multiple myeloma in 2016

Table 2 and Fig. 2 show the incidence and mortality for each of the 33 provinces in 2016. The ASIR were highest in Hong Kong Special Administrative Region, Macao Special Administrative region, and Shanghai, and were lowest in Gansu, Hainan, and Yunnan, respectively. The ASMR were highest in Hong Kong Special Administrative Region, Zhejiang, and Shanghai, and were lowest in Hainan, Fujian, and Shandong, respectively.

**Table 2:** Incidence and mortality of multiple myeloma by province of China in 2016

	Incidence		Mortality	
	Cases (thousands)	Rates (per 100,000)	Deaths (thousands)	Rates (per 100,000)
Anhui	0.53 (0.46–0.61)	0.75 (0.65–0.86)	0.43 (0.37–0.51)	0.62 (0.53–0.73)
Beijing	0.47 (0.30–0.56)	1.78 (1.12–2.11)	0.21 (0.13–0.26)	0.85 (0.55–1.05)
Chongqing	0.32 (0.29–0.39)	0.84 (0.75–1.00)	0.24 (0.20–0.30)	0.63 (0.53–0.77)
Fujian	0.33 (0.28–0.41)	0.82 (0.71–1.04)	0.21 (0.18–0.28)	0.55 (0.46–0.73)
Gansu	0.19 (0.17–0.23)	0.69 (0.59–0.80)	0.16 (0.14–0.20)	0.60 (0.51–0.72)
Guangdong	1.47 (1.10–1.73)	1.40 (1.06–1.62)	0.67 (0.53–0.79)	0.69 (0.55–0.81)
Guangxi	0.45 (0.39–0.54)	0.88 (0.76–1.05)	0.34 (0.28–0.42)	0.67 (0.57–0.84)
Guizhou	0.28 (0.23–0.31)	0.75 (0.62–0.83)	0.26 (0.21–0.31)	0.70 (0.59–0.83)
Hainan	0.07 (0.06–0.09)	0.73 (0.63–1.02)	0.05 (0.04–0.07)	0.53 (0.43–0.76)
Hebei	0.74 (0.62–1.09)	0.85 (0.73–1.27)	0.48 (0.39–0.69)	0.58 (0.47–0.84)
Heilongjiang	0.45 (0.40–0.60)	0.89 (0.78–1.18)	0.31 (0.27–0.41)	0.64 (0.55–0.83)
Henan	0.87 (0.75–1.19)	0.86 (0.75–1.18)	0.60 (0.51–0.82)	0.62 (0.53–0.83)
Hubei	0.79 (0.67–0.93)	1.12 (0.96–1.31)	0.44 (0.37–0.52)	0.65 (0.55–0.78)
Hunan	0.82 (0.61–0.93)	1.03 (0.77–1.16)	0.60 (0.47–0.70)	0.77 (0.59–0.88)
Inner Mongolia	0.27 (0.24–0.36)	0.92 (0.80–1.22)	0.17 (0.14–0.23)	0.62 (0.52–0.82)
Jiangsu	1.33 (1.15–1.64)	1.26 (1.10–1.55)	0.59 (0.50–0.74)	0.58 (0.49–0.72)
Jiangxi	0.46 (0.28–0.53)	0.98 (0.61–1.13)	0.36 (0.24–0.43)	0.80 (0.52–0.95)
Jilin	0.33 (0.28–0.42)	0.91 (0.80–1.18)	0.22 (0.19–0.27)	0.64 (0.55–0.80)
Liaoning	0.66 (0.58–0.80)	1.05 (0.91–1.24)	0.41 (0.34–0.50)	0.66 (0.56–0.81)
Ningxia	0.05 (0.04–0.06)	0.79 (0.69–0.91)	0.04 (0.03–0.05)	0.65 (0.55–0.77)
Qinghai	0.05 (0.04–0.06)	0.87 (0.74–1.04)	0.04 (0.03–0.05)	0.75 (0.63–0.92)
Shaanxi	0.37 (0.33–0.44)	0.84 (0.74–1.00)	0.27 (0.23–0.33)	0.63 (0.53–0.78)
Shandong	1.08 (0.91–1.59)	0.88 (0.74–1.29)	0.67 (0.55–0.96)	0.56 (0.46–0.81)
Shanghai	0.63 (0.31–0.79)	1.89 (0.90–2.35)	0.30 (0.16–0.39)	0.95 (0.48–1.22)
Shanxi	0.33 (0.28–0.44)	0.81 (0.70–1.11)	0.22 (0.18–0.31)	0.58 (0.48–0.80)
Sichuan	0.89 (0.77–1.01)	0.86 (0.75–0.97)	0.69 (0.59–0.85)	0.67 (0.57–0.82)
Tianjin	0.24 (0.20–0.31)	1.39 (1.18–1.79)	0.11 (0.09–0.14)	0.67 (0.56–0.85)
Tibet	0.02 (0.01–0.02)	0.81 (0.64–0.91)	0.02 (0.01–0.02)	0.80 (0.64–0.93)
Xinjiang	0.22 (0.19–0.30)	1.01 (0.88–1.39)	0.15 (0.13–0.21)	0.75 (0.64–1.02)
Yunnan	0.34 (0.31–0.41)	0.74 (0.67–0.87)	0.29 (0.25–0.37)	0.64 (0.55–0.81)
Zhejiang	1.22 (0.58–1.53)	1.76 (0.82–2.20)	0.67 (0.32–0.85)	1.01 (0.48–1.29)
Hong Kong*	0.27 (0.13–0.33)	2.31 (1.15–2.87)	0.13 (0.06–0.16)	1.07 (0.55–1.35)
Macao*	0.01 (0.01–0.02)	2.06 (1.18–2.80)	0.01 (0.00–0.01)	0.99 (0.57–1.31)

Data in parentheses are 95% uncertainty intervals

*Special Administrative Regions

**Fig. 2:** Age-standardized incidence rates (**a**) and mortality rates (**b**) of multiple myeloma for 33 provinces, 2016

### Trends in incidence and mortality of multiple myeloma from 2006 to 2016

As shown in Fig. 3, the ASIR of multiple myeloma increased significantly with an APC of 3.28 from 2006 to 2014 and 2.32 from 2014 to 2016. On the other hand, the ASMR increased from 2006 to 2014 with an APC of 0.78 and remained stable from 2014 to 2016 with an APC of 0.34.

**Fig. 3:** Trends in age-standardized incidence and mortality of multiple myeloma from 2006 to 2016 in China

## Discussion

The present study is the most comprehensive evaluation of the large and ever-growing burden of multiple myeloma in China. Due to the standardized methods for estimates of multiple myeloma metrics used in the GBD study, it is possible to compare incidence and mortality at province level in China. Based on the disparities in disease burden, different strategies for disease prevention and control should be employed when health policy is developed in the future.

The patterns of burden of MM varied by age and sex. Unlike most other cancers in China, MM was rare between 0–14 years old. Both incidence and mortality rate were increased with age in most of the age groups, which was consistent with previous study published by our group [4]. Notably, male predominance of incidence and mortality was seen in all age groups. According to the GBD study, both the age-standardized incidence and mortality rate in China were lower than global (ASIR was 1.93 per 100,000 population with 95% UI 1.87–2.19, ASMR was 1.37 per 100,000 population with 95% UI 1.26–1.52) and our neighbor Japan (ASIR was 2.18 per 100,000 population with 95% UI 1.91–2.78, ASMR was 1.30 per 100,000 population with 95% UI 1.17–1.58) [5, 7]. Geographical differences across provinces had an important role in the epidemiological characteristics of MM in China. Overall, higher incidence and mortality rates were seen in the clustered developed provinces, with 2–3-fold gap between those developed and less-developed provinces. In addition, the incidence level in the developed provinces was more close to those developed countries in Asia, like Japan. The low incidence and mortality rates in less-developed provinces may be associated with the poor medical accessibility. The heterogeneous pattern of epidemiological characteristics of MM across provinces highlighted the need to improve the access to health services leading to more precise diagnosis and early treatment, especially in those less-developed provinces.

Improving diagnosis and treatment techniques had a positive effect on the mortality of MM. The result of EUROCARE-5 [8] reflected the encouraging trend of MM and plasmacytoma with survival increase from 29.8% in 1997–1999 to 39.6% in 2006–2008. High-dose chemotherapy followed by autologous hematopoietic cell transplantation changed dramatically the perspective for young patients, while novel agents such as bortezomib, thalidomide, and lenalidomide prolonged the survival for both young and elderly patients [1]. Real-world study from the Swedish Myeloma Registry showed that the 5-year relative survival increased from 47.3% in the period of 2008–2010 to 51.3% in the period of 2011–2015 with the increased use of novel agents [9]. Another study from the Swedish Cancer Register also showed that the 10-year mortality in patients younger than 60 years in 1994–2003 reduced 29% compared with that in 1987–1993 [10]. A study from the Asian Myeloma Network, involving 3405 symptomatic MM patients, demonstrated that the median overall survival was 47 months (95% CI 44.0–50.0) and better survival was observed in those treated with stem cell transplantation or new drugs [11]. In a multicenter study [12] including 940 newly diagnosed MM patients from China, the median overall survival (OS) was 54 months with more survival benefit in IgG patients receiving bortezomib. Notably, the Food and Drug Administration of China approved bortezomib in 2005 and lenalidomide in 2013 for the treatment of MM. Until then, the Chinese patients had a chance of being exposed to novel drugs because they received treatment with many clinical trials in tertiary hospitals [11]. In our study, the mortality of MM increased from 2006 to 2014, but remained stable since 2014, regardless of the continuous increasing incidence. Similarly, a systematic analysis for global burden of MM [13] demonstrated that there was an improvement in age-standardized death rate form from 1990 to 2016 in high-income sociodemographic index regions despite increasing incidence rates, which indicated that patients with MM, especially in developed areas, benefited from treatment advancement. All these findings suggested modern risk-adaptive therapies brought longer survival for MM patients and then led to decrease of mortality of MM. There are marked differences in the epidemiological characteristics of MM between western and eastern countries. Increasing incidence trends were verified for most of the European and American countries, which was attributed to better accessibility to health services and more precise diagnosis of MM [14]. In Great Britain, the MM age-adjusted incidence per100,000 increased from 3.2 in 1975–1979 to 5.4 in 2005–2009. In addition, the data in this study argued strongly against the notion that environmental exposures were responsible for the changes in incidence [15]. In the USA, the incidence rates of MM per 100,000 remained stable over the three decades, with 4.6 in 1981–1990, 4.7 in 1991–2000, and 4.7 in 2001–2010, respectively [16]. In our study, we determined that the burden of MM was increasing in China during the past decade. This upward trend of incidence may be explained partly by some factors such as aging, better access to diagnosis, excess body weight [17], and occupational exposures [18], but much of this trend was largely unexplained and further study focused on etiology of MM should be performed.

The interpretation of our study has several limitations. First, all the general limitations described by the GBD collaboration group [5–7, 19] apply to the present study. Second, the low incidence and mortality rates of MM both in the national level and in the province levels may bias the estimated results using the standard GBD methodology. Third, population growth and changes of socioeconomic structures should also be taken into account; the spatial-temporal trends of MM burden needs to be interpreted cautiously.

## Conclusions

This is the first study to present spatiotemporal variation in MM burden in China nationally. Higher incidence and mortality rates were observed in males and older individuals with geographical differences across provinces. A significant increase in the incidence of MM was notable. The study results will be useful for policy-making with respect to disease prevention and the development of management strategies.

## Data Availability

The data that support the findings of this study are available from the Chinese Center for Disease Control and Prevention, but restrictions apply to the availability of these data, which were used under license for the current study, and thus are not publicly available. However, data are available from the authors upon reasonable request and with permission from the Chinese Center for Disease Control and Prevention.

## Abbreviations

APCs: Annual percentage changes
ASIR: Age-standardized incidence rates
ASMR: Age-standardized mortality rates
GBD: Global burden of disease
ICD: International classification of diseases
MM: Multiple myeloma
OS: Overall survival
UI: Uncertainty interval
